The article "High-dose radiation-induced immunogenic cell death of bladder cancer cells leads to dendritic cell activation" was published in 2024. Journal: PLoS One.

# High-dose radiation-induced immunogenic cell death of bladder cancer cells leads to dendritic cell activation

**DOI:** 10.1371/journal.pone.0307024

**Published:** 2024-09-04

**Authors:** Xianlin Zeng, Daiqin Luo, Shuai Zhang, Zhonghui Cui, Yun Wang, Jin Chen, Shichao Zhang, Lijing Teng, Zuquan Hu, Lina Liu, Shi Zhou, Zhu Zeng, Jinhua Long

**Affiliations:** 1 School of Biology and Engineering/School of Basic Medical Sciences, Guizhou Medical University, Guiyang, China; 2 Engineering Center of Cellular Immunotherapy of Guizhou Province, Guiyang, China; 3 Key Laboratory of Infectious Immunity and Antibody Engineering of Guizhou Province, Guiyang, China; 4 Department of Interventional Radiology, Affiliated Hospital of Guizhou Medical University, Guiyang, China; 5 Key Laboratory of Endemic and Ethnic Diseases, Ministry of Education, Guizhou Medical University, Guiyang, China; 6 State Key Laboratory of Functions and Applications of Medicinal Plants, Guizhou Medical University, Guiyang, China; 7 Department of Head and Neck, Affiliated Tumor Hospital of Guizhou Medical University, Guiyang, China; University of Illinois, UNITED STATES OF AMERICA

## Abstract

Radiotherapy is a commonly used method in the treatment of bladder cancers (BC). Radiation-induced immunogenic cell death (ICD) is related to the immune response against cancers and their prognoses. Even though dendritic cells (DC) act as powerful antigen-presenting cells in the body, their precise role in this ICD process remains unclear. Accordingly, an *in vitro* study was undertaken to ascertain whether high-dose radiation-induced ICD of BC cells could regulate the immune response of DC. The results indicated that high-dose radiation treatments of BC cells significantly increased their levels of apoptosis, blocked their cell cycle in the G_2_/M phase, increased their expression of ICD-related proteins, and upregulated their secretion of CCL5 and CCL21 which control the directed migration of DC. It was also noted that expression of CD80, CD86, CCR5, and CCR7 on DC was upregulated in the medium containing the irradiated cells. In conclusion, the present findings illustrate that high-dose radiation can induce the occurrence of ICD within BC cells, concomitantly resulting in the activation of DC. Such findings could be of great significance in increasing the understanding how radiotherapy of BC may work to bring about reductions in cell activity and how these processes in turn lead to immunoregulation of the function of DC.

## Introduction

Bladder cancers (BC) are among the most common tumors of the urinary system [1]. While radical cystectomy (RC) is the recommended treatment for BC, a loss of bladder function after RC not only reduces patient quality of life but also negatively affects the intestinal and reproductive functions of these individuals, and even increases the risk of post-operative deaths [2]. With a potential decrease in patient quality of life expectations and the occurrence of various complications from RC, bladder preservation therapy has gained significant interest from researchers who treat BC [3,4].

The article "High-dose radiation-induced immunogenic cell death of bladder cancer cells leads to dendritic cell activation" was published in 2024. Journal: PLoS One.

Radiotherapy is one important protocol used in BC preservation therapies. Radiotherapy not only directly kills tumor cells by damaging their DNA, it also leads to a blocking of their cell cycle, and an increased release of lethal reactive oxygen species/apoptosis. Interestingly, these events also can induce host immune responses against the cancer cells, primarily mediated by the activities of antigen-presenting cells (APC). Among these types of cells are the dendritic cells (DC) that ‘capture’ cancer antigens in the local microenvironment and process/present them to naïve T-cells residing in lymph nodes. This, in turn, leads to the proliferation of cancer antigen-specific T-cells [5,6] and an overall propagation of the host anti-tumor response.

Immunogenic cell death (ICD) is a form of regulated cell death that activates adaptive immunity [7]. This process enhances DC antigen presentation capacity in part through the release from cancer cells of danger-associated molecular patterns (DAMP) molecules, including high mobility group box 1 (HMGB1), calreticulin (CRT), heat shock protein 70 (HSP70) and adenosine triphosphate (ATP), that ultimately activate CD8^+^ T-cell adaptive responses [8]. HMGB1 can induce the maturation of DC and promote the processing/presentation of tumor antigens in association with surface major histocompatibility (MHC)-I molecules [9]. CRT can act as a signal to activate DC phagocytosis and promote antigen presentation ability; CRT can also act as an immunogenicity signal to recruit more DC to the tumor environments. HSP70 ‐ readily recognized by APC through CD91 molecules ‐ activates nuclear factor (NF)-κB signal pathways in the DC; the result of this activation is an enhanced formation/release of pro-inflammatory cytokines and activation of local inflammatory responses [10].

Some studies have shown that compared with conventional radiotherapy, high-dose radiation can induce cancer cell apoptosis and the release of more tumor cell immunogenic agents [11]. Other studies showed that high-dose radiation can also damage tumor blood vessels, making it easier for immune cells in the blood circulation to enter the tumor itself and perform immune responses against the target cells [12]. While radiotherapy is the main treatment employed for BC patients (with the goal of post-operative clearance of residual lesions and bladder preservation), how the high dose radiation-induced immune response works to bring about this positive outcome is still unclear. Accordingly, the *in vitro* study presented here sought to better define how ICD works against BC cells following high-dose radiation treatment as well as to examine the process of immune sensitization in the overall removal of these cancer cells.

The article "High-dose radiation-induced immunogenic cell death of bladder cancer cells leads to dendritic cell activation" was published in 2024. Journal: PLoS One.

## Materials and methods

### Cell culture

The BT-B human BC cell line was purchased from Fenghbio Corporation (Hunan, China), and authentication by short tandem repeat profiling. The cells were cultured in T-25 flasks containing complete RPMI-1640 medium (Gibco, Grand Island, NY) (RPMI 1640 supplemented with 10% fetal bovine serum [FBS; Biological Industries, Beit Hamek, Israel] and 100 IU/ml penicillin-streptomycin [Gibco]), and maintained in a humified 5% CO_2_ air incubator at 37°C. Cells were routinely passaged when they reached 90% confluence.

For use in the experiments outlined below, the BT-B cells (in logarithmic growth phase) were irradiated for 0, 109, 217, 543, or 977 sec with 160 kV, 24 mA X-rays at doses of 0, 2, 4, 10, or 18 Gy using an RS-2000 system (Rad Source Technologies, Atlanta, GA).

### Preparation of DC

Human peripheral blood mononuclear cells (PBMC) were isolated from the peripheral blood of healthy individuals who all had donated blood at the Guizhou Blood Center. All PBMC were isolated using standard protocols of density gradient centrifugation over lymphocyte separation medium [13]. After isolation from the interphase, the harvested cells were pooled and counted on a hemocytometer. The cells were diluted to 2×10^7^/ml with complete RPMI-1640 medium and then 1 ml aliquots of the cells were placed into T-75 flasks and allowed to adhere for 2 hr at 37°C. Thereafter, non-adherent cells were removed by decant-ing/gentle rinsing, and then all adherent cells were collected into a 15-ml centrifuge tube using a cell scraper. From the recovered cells, all CD14^+^ monocytes were isolated using immunomagnetic beads (Miltenyi Biotech, Teterow, Germany), following manufacturer protocols [14]. All protocols employed here were approved by the Ethics Committee of the Affiliated Hospital of Guizhou Medical University (#2020162, 2020/4/9). Healthy people were recruited from July 1, 2020, to October 23, 2023, and blood samples were obtained to isolate Human peripheral blood mononuclear cells. Verbal informed consent was obtained from each willing participant and noted using an electronic signature.

The isolated CD14^+^ monocytes were then cultured in T-75 flasks containing complete RPMI-1640 medium that was also supplemented with 150 ng/ml recombinant human granulo-cyte-macrophage colony-stimulating factor (rhGM-CSF) and 100 ng/ml recombinant human interleukin (IL)-4 (rhIL-4) (both from Peprotech, Cranbury, NY). These cells were maintained at 37°C for 5 days to allow for the induction of immature DC (imDC).

The article "High-dose radiation-induced immunogenic cell death of bladder cancer cells leads to dendritic cell activation" was published in 2024. Journal: PLoS One.

### DC were cultured with conditioned media of BT-B cells

After the X-ray treatment, the BT-B cells were collected from the flasks using cell scrapers and then counted. Aliquots containing 5×10^6^ irradiated BT -B cells were then placed into 6-well plates and cultured at 37°C for 48 hr. At that point, the culture media was collected and any cell debris present was removed by centrifugation at 100 ×g for 5 min (4°C), followed by filtration through a 0.22-μm membrane (Millipore, Boston, MA). This supernatant was then used to treat the imDC.

Specifically, imDC (generated as above) were harvested, counted, and suspended in complete RPMI medium, and aliquots containing 10^6^ imDC were placed into new 6-well plates with each well already containing 1 ml RPMI-1640/20% FBS. Immediately after seeding, 1 ml of the irradiated BT-B cell medium was then added to designated wells; negative control (NC) wells received phosphate-buffered saline (PBS, pH 7.4) in place of the BT-B medium. Other control groups consisted of 10^6^ imDC that received 1 ml “conditioned” media of non-irradiated BT-B cells ((0 Gy+DC) that was generated in parallel with the irradiated cells (i.e., 2 Gy+DC, 4 Gy+DC, 10 Gy+DC, 18 Gy+DC). All cells were then maintained at 37°C for 48 hr before being analyzed as outlined below.

### Cell cycle and apoptosis

After irradiation as above, BT-B cells were seeded at 2×10^6^ in 6-well plates and cultured for 48 hr. To evaluate cell cycle status in the cultures, the cells were then collected and fixed overnight with 95% ethanol; thereafter, the cells were centrifuged (100 ×g, 5 min), washed with PBS (three times), re-suspended in a solution of dye buffer containing 15 μl propidium iodide/ml (PI; 4A Biotech, Beijing, China), and incubated at room temperature for 15 min [15].

To assess levels of apoptosis in the cells, parallel 48-hr cultures of the cells were collected, centrifuged (100 ×g, 5 min), washed PBS (three times), and then re-suspended in a solution of Annexin V-FITC (Meilunbio, Beijing) dye. The samples were then incubated in the dark at 25°C for 30 min. PI dye was added 5 min before the flow cytometry was performed.

Both the cell cycle and apoptosis endpoints in the cells were then evaluated using a BD FACSCanto II flow cytometer (BD, Franklin Lakes, NJ) that employed associated FACSDiva software. A minimum of 10,000 events/sample was acquired each time. Statistical evaluations were performed obtained using software from Flowjo (Ashland, OR). All outcomes that are then presented are the results from three independent experiments.

The article "High-dose radiation-induced immunogenic cell death of bladder cancer cells leads to dendritic cell activation" was published in 2024. Journal: PLoS One.

### Reverse transcription-polymerase chain reaction

After irradiation as above, BT-B cells were cultured for 48 hr to collect BT-B cells. The imDC were cultured with conditioned media of BT-B cells for 48 hr, and then these DC were collected. The cells were then treated as below to assess the expression of ICD-related genes in the BC cells and of surface molecule genes in the DC populations. In each case, total RNA from the cells (2×10^6^ total cells/sample) was extracted using TRIzol (Invitrogen, Carlsbad, CA) using standard protocols [16]. The total RNA isolated was evaluated for quantity and quality using a NanoDrop Ultramicro spectrophotometer (ThermoFirsher Scientific, Waltham, MA). Based on the outcomes, aliquots containing 1 μg total RNA/sample were reverse-transcribed to cDNA using a Fast-king gDNA Dispelling RT Supermix (Tiangen, Beijing). The total reaction volume was always maintained at 20 μl. Real-time PCR was then performed using a SYBR Premix Ex Taq kit (Takara, Tokyo, Japan). The specific primers used are listed in Table 1. *GAPDH* was used as the internal reference gene in all cases; mRNA expression levels of each gene of interest were then calculated using the ΔΔCT method [17]. In the ultimate data analyses, the relative expression levels in the control cells were set as 1.

**Table 1:** Primers used in this study.

Gene	Primer sequences (5’ → 3’)
*GAPDH*	F: GACCTGACCTGCCGTCTA
	R: AGGAGTGGGTGTCGCTGT
*BAK1*	F: GGACGACATCAACCGACGCTATG
	R: AACAGGCTGGTGGCAATCTTGG
*CRT*	F: AGATAAAGGTTTGCAGACAAGC
	R: CATGTCTGTCTGGTCCAAACTA
*Casp-1*	F: TTGAAGGACAAACCGAAGGTG
	R: GTGGAAGAGCAGAAAGCGATAA
*Casp-3*	F: GGAACAAATGGACCTGTTGAC
	R: CTCAATGCCACAGTCCAGTTC
*HMGB-1*	F: AAATGAAAACCTATATCCCTCCC
	R: GGGCGATACTCAGAGCAGAAG
*HSP70A1A*	F: GACTCCCGTTGTCCCAAG
	R: CGGTTCCCTGCTCTCTGT
*CD80*	F: GTGGTCACAATGTTTCTGTTGA
	R: GTTCTTGTACTCGGGCCATATA
*CD86*	F: TGCTCATCTATACACGGTTACC
	R: TGCATAACACCATCATACTCGA
*HLA-DR*	F: CCAGAGACTACAGAGAATGTGG
	R: TTGATGATGAAGATGGTCCCAA
*CCR5*	F: GCAGCTCTCATTTTCCATACAG
	R: GACACCGAAGCAGAGTTTTTAG
*CCR7*	F: AGACCATGACCGATACCTACC
	R: GCAAAAGTGGACACCGAAGA
*CD11c*	F: AGCAGCCACGAACAATTCAC
	R: GAGACCTCCACATCCATCCA

### Western blot

The BT-B cells were irradiated as above and then cultured for 48 hr. The cells were then collected and total proteins from the cells were extracted using a RIPA cell lysis solution (R0010) containing PMSF (P0100) (both Solarbio, Beijing). After clearing debris by centrifugation, the lysate was evaluated for total protein content using a BCA kit (Solarbio). An aliquot containing 50 μg of total protein was then loaded into a 12% SDS-PAGE gel; to permit subsequent localization of the proteins of interest separate wells on the gel were loaded with a standard of each protein of interest. The sample proteins were then resolved and electrotransferred to a nitrocellulose membrane (Millipore, Boston, MA). The membrane was incubated at 25°C for 1 hr in a solution of 5% skim milk powder-TBST (TBS buffer [pH 7.4] containing 0.1% Tween-20) to block non-specific binding sites. After three washes with TBST, the membrane was placed in a solution of TBST containing specific antibodies against rabbit anti-human GAPDH (10494-1-AP; Protein-tech, Rosemont, USA), HMGB1 (D260488; BBI, Shanghai, China), CRT (AB92516; Abcam, Cambridge, UK), and HSP70 (AB181606, Abcam, Cambridge, UK). Levels/dilutions of each antibody used were recommended by the various manufacturers. The membrane was then incubated overnight at 4°C with gentle rocking. After three gentle rinses with TBST, the membrane was placed in a solution of TBST containing horseradish peroxidase-conjugated anti-rabbit IgG (ZB-2306; ZSGB-BIO, Beijing) and incubated at room temperature for 1 hr. After final gentle rinsing with TBST (three times), protein bands were visualized using an enhanced chemiluminescence (ECL) kit (Beyotime, Beijing). In all cases, GAPDH served as the internal reference protein. Experiments were repeated three times with three triplicates for each experiment. Expression levels for each protein of interest were based on densitometric scanning of each band after alignment with its corresponding standard. All analyses were performed using Image J software (NIH, Bethesda, MD).

The article "High-dose radiation-induced immunogenic cell death of bladder cancer cells leads to dendritic cell activation" was published in 2024. Journal: PLoS One.

### Enzyme-linked immunosorbent assay (ELISA)

Specific antibody-coated ELISA plates for the measurements of human CCL5, CCL21 (4A Biotech, CHE0092, CHE0140), HSP70, HMGB1, and CRT (ZK-H182, ZK-H1377, ZK-H760) were purchased from Zikerbio (Shenzhen, China). For assays of each isolated lysate sample from the BC cells (see above), 100 μl kit standard or of the samples were added to the dedicated wells in corresponding plates, and the materials were then covered and incubated for 90 min at 37°C. After removal of the well contents and gentle washing with kit-provided wash buffer (three times), 100 μl kit biotin-antibody diluent was added to each well and the plates were incubated for a further 60 min at 37°C. After four washes with kit buffer, enzyme binding diluent (100 μl) was added to each well and the plate was incubated for 30 min at 37°C. After a final four washes with buffer, kit chromogenic solution (100 μl) was added to each well and the plate was incubated in the dark for 20 min at 37°C. After the addition of 100 μl Stop Reagent to the wells, the absorbance value at 450 nm in each well was assessed using an Imark microplate reader (BioRad, Hercules, CA). Levels of each indicated protein in the test samples were calculated by extrapolation from standard curves generated in parallel using kit-provided standards. Each experiment was repeated three times, with three triplicates for each regimen evaluated.

The article "High-dose radiation-induced immunogenic cell death of bladder cancer cells leads to dendritic cell activation" was published in 2024. Journal: PLoS One.

### ATP measurement

Extracellular secretion of ATP by the BC cells was evaluated using an ATP kit (A095-2-1, Nanjing Jiancheng Bioengineering, Nanjing, China), according to manufacturer protocols. In brief, BT-B cells were irradiated, collected, counted, seeded into 6-well plates (at 10^6^/well), and cultured at 37°C for 48 hr. At that point, culture supernatants were collected and ATP levels were measured with the kit. Each experiment was repeated three times, with three triplicates for each experimental condition.

### Immunofluorescence

Briefly, imDCs were fixed with 4% PFA and permeabilized with 0.1% Triton X-100. The cells were incubated with anti-CD11c rabbit antibody (97585S; CST, Massachusetts, USA) overnight at 4°C, and cells were counterstained with Alexa 488 anti-rabbit IgG (R37116, ThermoFisher, Waltham, USA) for 1 hour at room temperature in the dark. The cytoskeleton (actin filaments) was stained with rhodamine phalloidin (ab235138, Abcam, Cambridge, UK) for 30 minutes and nuclei were stained with DAPI (4,6-diamidino-2-phenylindole, Solarbio, Beijing, China) for 5 minutes. Images were obtained with an Olympus fluorescence microscope.

### Statistical analyses

All data are expressed as the mean ± SD from at least three independent experiments. All data was checked to meet the Shapiro-Wilk normality test. Statistical comparisons between the treatment groups were made using a Student’s *t*-test. A p-value < 0.05 was considered significant. Data analyses were all performed using Prism software (v.7.0, GraphPad, San Diego, CA); images were analyzed using Image J software.

## Results

### High-dose radiation promoted apoptosis among BT-B cells

After normal culture for 48 hr, the apoptosis of BT-B cells was closely related to the radiation dose (Fig 1). Compared with the non-irradiated group (0 Gy), a change in the number of apoptotic cells among the BT-B cells treated with 2 Gy and 4 Gy radiation was not a significant difference. In comparison, a significant difference in apoptosis of BT-B cells was observed with the 10 Gy dose, with apoptotic cells accounted for 11.4% of the total cell numbers, which is the proportion in the Q2 quadrant of the cross gate in Fig 1A. Interestingly, the number of apoptotic cells in BT-B cells irradiated by 18 Gy radiation accounted for just 7.7% of the total cells (Fig 1A). To validate these outcomes, some apoptosis marker proteins were evaluated (Fig 1C). It was found that the gene expressions of several apoptosis-related proteins Casp-1, Casp-3, and BAK1 were up-regulated after the BT-B cells received higher radiation levels.

The article "High-dose radiation-induced immunogenic cell death of bladder cancer cells leads to dendritic cell activation" was published in 2024. Journal: PLoS One.

**Fig 1:** Apoptosis in irradiated BT-B cells. (A) Apoptosis levels in cells after 0, 2, 4, 10, or 18 Gy exposures were analyzed by flow cytometry. The density of cells is shown by various colors in the picture. Each cell is a small blue dot, and the color shifts from blue to red, indicating that the cell density is gradually increasing. (B) Relative levels of apoptosis (Fold change related to 0 Gy). (C) mRNA expression levels of apoptosis-related proteins Casp-1, Casp-3 and BAK1 in the cells. Data from n  =  6 biologically independent samples. NS p > 0.05, *,**,***p < 0.05, < 0.01, < 0.001.

### High-dose radiation impact on cell cycle with the BT-B cells

Changes in the cell cycle progression within BT-B cells appeared to follow a dose-related relationship with the level of radiation used for treatment (Fig 2). Specifically, with a rise in radiation dose, both the proportion of BT-B cells in the G_2_/G_1_ phase increased and those staying in the G_2_ phase increased significantly. Among BT-B cells that were not irradiated, only about 19.8% of the cells stayed in the G_2_ phase, which is the proportion of G_2_ phase cells represented by the blue part in the lower part of Fig 2A. In comparison, after 18 Gy radiation, 62.6% of the BT-B cells remained in the G_2_ phase (The detailed data are shown in the Excel file of the cell cycle S1 Table in S1 Data).

**Fig 2:** Cell cycle in irradiated BT-B cells. (A) Cycle status of cells after 0, 2, 4, 10, or 18 Gy exposures were analyzed by flow cytometry. (B) Relative percentages of cells in the G_2_/G_1_ phase. Data from n  =  6 biologically independent samples. NS p > 0.05, *p < 0.05, ** < 0.01.

### Immunogenic cell death (ICD) of BT-B cells induced by radiation

Immunogenic death of cancer cells occurs with the release of risk associated molecular pattern (DAMP) molecules, including high mobility group box 1 (HMGB1), calreticulin (CRT), heat shock protein 70 (HSP70), and adenosine triphosphate (ATP). Levels of signature proteins for ICD were evaluated at both the mRNA and protein levels. It was found that the gene expression levels of *HMGB1* and *CRT* in BT-B cells rose to their highest after the 4 Gy radiation (Fig 3A). The levels of HSP70, HMGB1, and CRT released into the culture medium were also increased by treatment of the BT-B cells with high-dose radiation (Fig 3B). Expression levels of HSP70 and HMGB1 were most elevated by the 10 Gy radiation (Fig 3C). The analyses here also noted that this treatment also caused significant elevations in the levels of ATP released into the culture medium (Fig 4). The ATP content in supernatants of the BT-B cultures (non-irradiated group) was only 15.64 nM; in comparison, cells irradiated with 10 Gy radiation had supernatant ATP levels of 38.03 nM. Lower radiation doses yielded far less impact on the expression of this marker.

The article "High-dose radiation-induced immunogenic cell death of bladder cancer cells leads to dendritic cell activation" was published in 2024. Journal: PLoS One.

**Fig 3:** Select ICD-related proteins in irradiated BT-B cells. (A) mRNA expression of HSP70A1A, HMGB1 and CRT. (B) Concentration of HSP70, HMGB1, and CRT in conditioned medium. (C) Protein expression levels of HSP70, HMGB-1, and CRT. (D) Western blotting. Data from n  =  6 biologically independent samples. NS p > 0.05, *,**,***,****p < 0.05, < 0.01, < 0.001, < 0.0001.

**Fig 4:** ATP release from BT-B cells irradiated with different doses of X-ray. Data from n  =  6 biologically independent samples. *p < 0.05.

### High-dose radiation impact on BT-B cell secretion of CCL5 and CCL21

DCs can migrate along a concentration gradient of CCL5 and CCL21 to reach lesions and lymph nodes. Therefore, the secretion level of CCL5 and CCL21 was measured to verify whether bladder cancer cells could induce the recruitment of DCs after radiotherapy in this study. After the irradiation treatments, it was also seen that the levels of CCL5 and CCL21 in the BT-B cell culture medium increased in tandem with the levels of radiation employed (Fig 5). For example, it was seen here that high-dose radiation increased measured levels of CCL5 released by the cancer cells (0, 10, and 18 Gy regimens resulted in culture levels of 1912, 2430, and 2412 pg CCL5/ml, respectively). Interestingly, conventional dosing (i.e., 2 Gy) resulted in suppressed CCL5 secretion, i.e., CCL5 secretion by BT-B cells was now 1122 pg CCL5/ml. With CCL21, this 10 Gy radiation exposure resulted in levels of concentration was 89.71 pg CCL21/ml. Lower radiation doses yielded far less impact on the expression of these markers. In comparison, control cell levels of just 56 pg CCL21/ml were observed in parallel. The study here saw that high-dose radiation increased the secretion levels of CCL5 by the cancer cells, while conventional doses of radiation suppressed CCL5 secretion.

**Fig 5:** The concentration of BT-B cells chemokines as a function of different radiation doses. The concentration of (A) CCL5 and (B) CCL21in a conditioned medium. Data from n  =  6 biologically independent samples. *,**,***,****p < 0.05, < 0.01, < 0.001, < 0.0001.

The article "High-dose radiation-induced immunogenic cell death of bladder cancer cells leads to dendritic cell activation" was published in 2024. Journal: PLoS One.

### Medium from BT-B cells irradiated with high-dose radiation affected imDC maturation

Since CRT and HMGB1 secreted by BT-B cells promote DC maturation, meanwhile chemokines secreted by BT-B recruit DC cells. Therefore, this research evaluated if the radiation treatment of the bladder cancer cells could affect the immunity function of DCs by detecting the expression levels of costimulatory molecules *CD80* and *CD86*, chemokine receptors *CCR5* and *CCR7*, antigen presentation related molecule HLA-DR and DC signature marker *CD11c* in imDC incubated for 48 hr with the medium derived from the irradiated cells. First, dendritic cells were identified in this research. As shown in Fig 6A, the cells highly expressed CD11c protein and had many short dendritic protrusions, indicating that the cells isolated in this study were dendritic cells. The results showed that the expression of *CD80*, *CD86*, and *CCR7* were all up-regulated and that of *HLA-DR* down-regulated when high-dose radiation was first used to treat the BT-B cells (Fig 6B). Notably, the expression of *CD80* and *CD86* in DC cells in the 10 Gy+DC group was threefold higher than that in the negative control group. Combining the results of bladder cancer cell apoptosis (Fig 1A), HMGB1 protein expression (Fig 3C), and chemokine CCL21 secretion (Fig 5) in this paper, it can be hypothesized that BT-B cells received the highest radiation dose of 10 Gy have the maximal effect on imDC.

**Fig 6:** Expression levels of genes for DC surface molecules after DC treatment with conditioned media of irradiated BT-B cells. (A) Immunofluorescence staining of imDC. Nuclei were stained with DAPI (blue), cytoskeleton with F-actin (red), and DC marker with CD11c (green). (B) The mRNA expression levels of *HLA-DR*, *CD11c*, *CD80*, *CD86*, *CCR5*, and *CCR7* in DC after 48 hr culture. In the statistical graph, NC = control group (DC without conditioned BT-B cell media). 0 Gy+DC = DC cultured with media of BT-B cells without radiation treatment. Various radiation doses used to treat BT-B cells prior to isolation of their media to then treat DC cells are noted: 2, 4, 10, and 18 Gy. Data from n  =  6 biologically independent samples. NS p > 0.05, *,**,***,****p < 0.05, < 0.01, < 0.001, < 0.0001.

## Discussion

With the continuous improvements in radiotherapy technology, the survival rate and quality of life of patients with bladder cancer (BC) have been enhanced [18]. At the same time, the application of radiotherapy in BC provides an alternative treatment for patients who do not want to accept cystectomy, and also for elderly patients who cannot undergo surgical resection [19]. However, the 2-year survival rate for older patients receiving radiation therapy is still only 42% [20]. Recent studies found that receiving a higher radiation dose was associated with improved overall survival in BC patients [21]. Conventional dose radiation was defined as being delivered at 1.8–2.0 Gy per fraction. High dose radiation was defined as delivered at > 2 Gy per fraction [22]. In addition, Peng et al. [23] found that BC-bearing mice that expressed anti-tumor GM-CSF and IL-21 had a higher number of CD8^+^ T-cells and significantly smaller tumor sizes after receiving radiation compared to mice that went untreated. Meanwhile, clinical studies have found that radiation-induced higher immune infiltration improved overall survival in patients with muscle-infiltrating BC [24]. Based on all of these cited papers, one could infer that radiation dose and the immune response induced by radiotherapy are important factors in the treatment of BC, but even so, the mechanisms underlying any radiation-induced immune responses against BC remain unclear. Accordingly, this study was undertaken to try to explore mechanisms underlying radiation-induced anti-tumor immunity, from the aspect of the killing effect of high-dose radiation on BC cells as well as the subsequent potential activation of DC induced by this type of BC cell treatment.

The article "High-dose radiation-induced immunogenic cell death of bladder cancer cells leads to dendritic cell activation" was published in 2024. Journal: PLoS One.

In this study, it was seen that the apoptosis among BT-B (BC) cells was the most significant difference after use of a 10 Gy radiation dose (Fig 1B). Among the various mechanisms known to be related to apoptosis, an increase in cell caspase-1 promotes programmed cell death by activating the production of both interleukin (IL)-1β and IL-18 [25,26]. Caspase-3 directly cleaves cellular proteins, such as cytoskeletal proteins and proteins needed for repairing DNA, resulting in cellular apoptosis [27,28]. Unlike the caspases, BAK1 promotes apoptosis by causing a reduction in cell membrane potential and the release of cytochrome C [29,30]. The current study found that the expression of caspase-1, caspase-3, and BAK1 all increased after high-dose radiation treatment and that these changes paralleled those seen in the frequency of apoptosis as detected by flow cytometry (Fig 1C). Concurrently, a dose-related relationship between changes in BT-B cell cycle progression and radiation dose was also noted. It was seen that with the higher radiation doses tested, the number of BC cells that stalled at the G_2_ phase increased significantly (Fig 2), indicating cell cycle progression was blocked at the G_2_/M checkpoint. Since radiotherapy can damage DNA, it can be inferred that due to DNA damage, BT-B cells were arrested in the G_2_ phase and could not enter the M phase for mitosis after radiotherapy, thus inhibiting cell proliferation [31,32].

The article "High-dose radiation-induced immunogenic cell death of bladder cancer cells leads to dendritic cell activation" was published in 2024. Journal: PLoS One.

Traditional radiation studies focus on its ability to damage DNA; however, recent studies show that a key mechanism driving the efficacy of radiation *in vivo* is an immune response triggered in/by irradiated tissues or cancer cells [33]. HSP70, HMGB1, CRT, and ATP are four representative markers of ICD [7]. Savage et al. [34] showed that the expression of CRT and HMGB1 increased in tumor tissues of mice after high dose radiation in breast cancer, enhancing tumor immunogenicity, much as what had been seen earlier in Golden et al. [35]. The current study also found that the expression of HSP70, HMGB1, and CRT by the BT-B cells after high-dose radiation exposure were all far greater than those seen after low-dose/no radiation exposure (Fig 3).

Interestingly, each of these proteins may impact the activities of cells involved in immune responses. For example, HSP70 can be rapidly recognized by APC through their CD91 surface receptors; this interaction promotes APC release of pro-inflammatory cytokines and triggers a Th17 cell-centered response [10,36,37]. HMGB1 is a histone-chromatin binding protein released after tumor cells are damaged by radiation and undergo apoptosis [38]. HMGB1 can also bind to toll-like receptors (TLR)-4 and -9 to up-regulate expression levels of DC immunophenotype molecules and promote DC maturation [9,39,40]. Lastly, CRT exposure on the cell surface can act as a DC phagocytosis signal, promote DC recruitment, and enhance DC antigen phagocytosis and presentation ability [41,42]. Even more, the extracellular ATP molecules that are released by dying cells (including the irradiated BC here) are known to be able to sensitize DC through the activation of P2X and P2Y ATP receptors on these APC [43]. The observations here of increased expression of HSP70, HMGB1, and CRT in conjunction with the increased release of ATP by the BC cells after high-dose radiation indicated to us that there was the occurrence of ICD among the BC cells due to the radiation (Fig 4). Such an outcome has clear potential implications for local DC in hosts who undergo radiation therapies to treat their BC.

An occurrence of ICD can induce local DC to mature and infiltrate into tumor tissues as part of an overall activation of host anti-tumor immune responses [44–46]. To ascertain if the high-dose radiation regimen here may have induced changes in the studied DC, the present study evaluated the concentrations of select DC chemokines CCL5 and CCL21 and expression levels of DC immunophenotype molecules after culturing imDC with these culture supernatants collected from irradiated BT-B cells. The study here saw that high-dose (10 Gy) radiation increased the release of CCL5 by the BC cells, i.e., CCL5 secretion by BT-B cells reached 2430 pg/ml after exposure to 10 Gy radiation. These outcomes are somewhat in contrast to those of Gawłowska-Marciniak and Niedzielski [47] and Tianyi and Zhiyuan [48] who noted that concentrations of CCL5 in the kidney tissues of healthy (non-radiation-exposed) adults (97.51 pg/ml) and in supernatants of peripheral nerve cell cultures (359.2 pg/ml). At the same time as the changes in the release of CCL5 by the BC cells, the radiation was also seen to cause an increase in the release of CCL21 by these irradiated cells (with maximum again being attained after the highest [10 Gy] radiation dose was used). This showed that BC cells after high-dose radiation exposure were somehow triggered to increase their release of CCL5 and CCL21 to recruit more DC (Fig 5). Because normal cells and unirradiated bladder cancer cells secrete very low levels of CCL5, they cannot recruit enough dendritic cells to initiate the immune response. This suggests that treating bladder cancer cells with high doses radiation may be an effective way to boost the immune response.

The article "High-dose radiation-induced immunogenic cell death of bladder cancer cells leads to dendritic cell activation" was published in 2024. Journal: PLoS One.

When they receive antigenic stimulation, imDC gradually differentiates into mature DC that display increased expression of co-stimulatory CD80 and CD86 molecule as well as the chemokine receptor CCR7. Once these expressions are all up-regulated, DC migration to secondary lymphoid tissues then occurs along chemotactic gradients associated with CCL21 (as well as with CCL19) [49]. In the present study, CD80, CD86, and CCR7 expressions by the imDC were most significantly increased after treatment with the conditioned media from high-dose radiation treated BT-B cells (Fig 6). Among them, increased expression of CD80 and CD86 indicates that the antigen presentation ability of DCs is improved, whereas increased expression of CCR7 indicates that DCs are better able to accept the chemokine CCL21 induction and then migrate to the lesion, reflecting the improved migration ability of DCs indirectly. This is consistent with the findings of Kulzer et al. [50] who found that treatment of colorectal cancer cells with 5 Gy radiation led to DC maturation [50,51]. In light of the observed increases in CCL5 and CCL21 expression when the culture medium of irradiated BC cells was used to treat imDC, it would appear that BC cells ‐ after high-dose radiation treatment were very impactful on the eventual maturation of DC and their invasive capacities/potentials. Such changes, if they occur *in situ/in vivo*, could have important implications for host health and long-term survival.

The article "High-dose radiation-induced immunogenic cell death of bladder cancer cells leads to dendritic cell activation" was published in 2024. Journal: PLoS One.

## Supporting information

S1 Data (RAR)
